This article has been retracted.

# Acellularized spinal cord scaffolds incorporating bpV(pic)/PLGA microspheres promote axonal regeneration and functional recovery after spinal cord injury

**DOI:** 10.1039/d0ra02661a

**Published:** 2020-05-18

**Authors:** Jia Liu, Kai Li, Ke Huang, Chengliang Yang, Zhipeng Huang, Xingchang Zhao, Shiqiang Song, Taisen Pang, Jing Zhou, Yuhai Wang, Chong Wang, Yujin Tang

**Affiliations:** Department of Orthopedics, Affiliated Hospital of Youjiang Medical University for Nationalities 18 Zhongshan II Road Baise Guangxi 533000 China tangyujin1967@163.com +86-0776-2833076; Academy of Orthopedics, Guangdong Province, The Third Affiliated Hospital of Southern Medical University Guangzhou Guangdong 510000 China; Department of Anatomy, Youjiang Medical College for Nationalities Baise Guangxi 533000 China; Academy of Orthopedics, People's Hospital of Ningxia Hui Autonomous Region Ningxia 502213 China; School of Mechanical Engineering, Dongguan University of Technology No. 1 University Road, Songshan Lake Dongguan Guangdong 523808 P. R. China wangchong@dgut.edu.cn +86-1341-6885162

## Abstract

Spinal cord injury (SCI) is a traumatic injury to the central nervous system (CNS) with a high rate of disability and a low capability of self-recovery. Phosphatase and tensin homolog (PTEN) inhibition by pharmacological blockade with bisperoxovanadium (pic) (bpV(pic)) has been reported to increase AKT/mTOR activity and induce robust axonal elongation and regeneration. However, the therapeutic effect of bpV(pic) in treating SCI is limited due to the lack of efficient delivery approaches. In this study, a composite scaffold consisting of an acellular spinal cord (ASC) scaffold and incorporated bpV(pic) loaded poly (lactic-*co*-glycolic acid) (PLGA) microspheres was developed, in order to improve the therapeutic effect of bpV(pic) on SCI. The inhibition of PTEN activity and activation of the mTORC1/AKT pathway, the axonal regeneration and the markers of apoptosis were analyzed *via* western blot and immunofluorescence *in vitro*. The bpV(pic)/PLGA/ASC scaffolds showed excellent biocompatibility and promoted the viability of neural stem cells and axonal growth *in vitro*. Implantation of the composite scaffold into rats with hemi-sectioned SCI resulted in increased axonal regeneration and functional recovery *in vivo*. Besides, bpV(pic) inhibited the phosphorylation of PTEN and activated the PI3K/mTOR signaling pathway. The successful construction of the composite scaffold improves the therapeutic effect of bpV(pic) on SCI.

## Abstract 2

Spinal cord injury (SCI) is a traumatic injury to the central nervous system (CNS) with a high rate of disability and a low capability of self-recovery.

## Introduction

Spinal cord injury (SCI), a serious traumatic injury to the spinal cord and central nervous system, is a major cause of motor disability and death.^1,2^ It is associated with limited functional recovery, mainly due to the limited endogenous regeneration capacity of host spinal cord tissue.^3,4^ SCI causes severance of axons and death of neurons, which lead to permanent functional impairments.^5,6^ The pathophysiology of acute SCI consists of both primary and secondary injuries. Secondary injury spreads from the primary injury site causing further tissue loss and dysfunction as well as a cascade of biological stress responses.^7^ Restricting the development of secondary injury and enhancing the intrinsic growth ability of neurons, which naturally declines during development, bears the possibility to improve functional recovery after SCI.^8,9^ Current therapeutic strategies for SCI include surgical decompression and pharmacotherapy.^10–12^ However, due to the limited understanding of the mechanisms involved in SCI progression, there is no effective strategy for treating this clinical challenge. Thus, there is an urgent need to develop superior approaches to improve the tissue regeneration and functional recovery after SCI.

PTEN is a well-characterized tumor suppressor gene that negatively regulates the PI3K–AKT–mTOR signaling pathway.^13^ The PI3K–AKT–mTOR pathway plays a critical role in regulating axon formation and extension.^14–17^ For instance, constitutively active AKT in embryonic chick dorsal root ganglion neurons increases axon branching, cell hypertrophy and growth cone expansion.^18^ Downstream of AKT is the mechanistic target of rapamycin (mTOR), a key factor in an intracellular signaling pathway that regulates protein synthesis, cell growth, proliferation, apoptosis and autophagy.^19^ mTOR is a component of the PI3K pathway and is directly phosphorylated by AKT, with phosphorylated mTOR acting as a central controller.^20^ Given that PTEN negatively regulates PI3K–AKT–mTOR activity by dephosphorylating phosphoinositide substrates, PTEN suppression likely increases axon growth by enhancing the activity of the PI3K–AKT–mTOR signaling cascade.^21^

PTEN inhibition by a number of approaches, including genetic deletion in mice, knockdown by shRNA, or pharmacological blockade by phosphatase inhibitors or selective antagonist peptides, leads to increased AKT/mTOR activity and robust axonal elongation and regeneration.^21,22^ Recently, several studies reported that [bpV(pic)], an inhibitor of PTEN, is able to activate the AKT/mTOR signaling pathway, thereby effectively enhancing the intrinsic growth capacity of axons.^23^ Importantly, bpV(pic) is able to protect nerve tissues following trauma, ameliorate secondary injury and promote neural stem cells (NSCs) differentiation into neurons, hence possessing tremendous potential to treat SCI.^24–26^

Herein, bpV(pic) encapsulated PLGA microspheres were produced in order to achieve a controlled release of bpV(pic) at the site of spinal cord injury. The presence of bpV(pic)/PLGA microspheres in the culture medium resulted in a promotion of axonal growth *in vitro*. Furthermore, we incorporated the bpV(pic)/PLGA microspheres into an acellular spinal cord (ASC) scaffold, and implanted the composite scaffold into a rat model with hemi-sectioned SCI *in vivo*, and attained the highest level of axonal regeneration and functional recovery compared to any other treatment conditions *in vivo*. We also confirmed that bpV(pic) was able to inhibit the phosphorylation of PTEN, leading to substantial activation of the mTORC1/AKT pathway. This led to decreased apoptosis, increased proliferation and axonal growth, and an overall ameliorated SCI recovery process.

## Materials and methods

### Preparation of bpV(pic)/PLGA microspheres

PLGA microspheres were prepared using the water-in-oil-in-water (w/o/w) double emulsification-evaporation technique. Precisely, 25 mg bpV(pic) and 25 mg of PVA were dissolved in 0.4 ml of deionized (DI) water. Afterwards, bpV(pic) aqueous solution was added into 4 ml of PLGA/dichloromethane solution (2.5%, w/v) dropwise, followed by magnetic stirring at 2000 rpm to form bpV(pic)/water/PLGA/DCM water-in-oil emulsions. Then, the water-in-oil emulsion was injected, while stirring, into a 40 ml aqueous solution of PVA (2% w/v). To prevent sedimentation of the polymer, the stirring speed was kept at 250 rpm. About 3 s after the injection, the stirring speed was slowly increased to 600 rpm. After emulsification for 5 min, the mixture was poured into 450 ml of distilled water with vigorous agitation. Then, the solvent was allowed to evaporate at room temperature with constant stirring and reduced pressure for 4–6 h to form the microspheres. Afterwards, the microspheres were centrifuged and washed several times so as to remove any residual PVA. After cryo-drying in a freeze-dryer (ALPHA2-4, Germany) for 48 h, bpV(pic)/PLGA microspheres in white powder form were obtained, and were stored in a dryer at room temperature.

### Fabrication of ASC scaffold

Adult Sprague Dawley (SD) rats were sacrificed by intraperitoneal injection with 10% chloral hydrate (60 ml kg^−1^). The thoracic spinal cords were harvested. The chemical extraction for ASC preparation was based on a previously described procedure.^35^ Briefly, thoracic spinal cords were treated with a series of detergents including DI water, Triton X-100 and sodium deoxycholate solution. Afterwards, all samples were rinsed using DI water and subsequently freeze-dried for 48 h in a freeze dryer and further sterilized by irradiation (5 kGy) with Co^60^ gamma ray before being used. All animal experiments were approved by the local ethics committee for animal research at Youjiang Medical College for Nationalities, and were performed in accordance with international standards for animal welfare.

### Fabrication of bpV(pic)/PLGA microsphere loaded ASC scaffolds

5 mg of bpV(pic)/PLGA microspheres were homogeneously dispersed in 200 μL of DI water *via* 5 min of ultra-sonication within a ultrasonic clean machine. The bpV(pic)/PLGA microsphere suspension was then added onto the ASC scaffold dropwise. Afterwards, the ASC scaffold adsorbed with bpV(pic)/PLGA microspheres were frozen at −80 °C and put into a freeze drier for 48 h to remove water, hence forming ASC scaffold incorporated with bpV(pic)/PLGA microspheres. To study the loading amount of bpV(pic) in PLGA microspheres, the content of bpV(pic) extracted from PLGA microspheres was measured. Typically, 50 mg of bpV(pic)/PLGA microspheres was dissolved in 2 ml of chloroform. Afterward, 0.5 ml of DI water was added into the bpV(pic)/PLGA/chloroform solution and subjected to 5 min of high speed vortex stirring and 20 min of centrifugation at 10 000 rpm. Till now, bpV(pic) could be extracted from the PLGA microspheres and dissolved in the aqueous phase. Then the concentration of bpV(pic) can be measured by reversed phase high performance liquid chromatography. The encapsulation efficiency of bpV(pic) in PLGA microspheres can be calculated as follows: encapsulation efficiency (EE, %) = the amount of bpV(pic) extracted from 50 mg of PLGA microspheres/total amount of bpV(pic) used for making 50 mg of PLGA microspheres. After calculation, in our study, 5 mg of bpV(pic) was incorporated in 100 mg of PLGA microspheres and the EE value of bpV(pic) in PLGA microspheres is 20.0%. As the mass ratio between bpV(pic) microspheres and ASC scaffolds is 10 : 90, 0.5 mg of bpV(pic) was encapsulated in 100 mg of PLGA/ASC composite scaffolds.

### Cell culture

The rat neural stem cell (NSC) was obtained from Cyagen Biosciences (Cat No. RASNF-01001, Suzhou, China). The cells were maintained in the NSC growth medium (Cat no. RASNF-90081, Cyagen Biosciences, Suzhou, China) at 37 °C in a 5% CO_2_ humidified incubator, with the supplemental of 1% penicillin–streptomycin, 2% B27, 20 ng ml^−1^ epidermal growth factor (EGF) and 10 ng ml^−1^ basic fibroblast growth factor (bFGF). For neurogenic differentiation, NSCs were plated in 6-well tissue culture plates coated PLL/laminin at 2 × 10^4^ cells per cm^2^ in with growth medium volume of 2 ml per well, and cells were incubated at 37 °C in a 5% CO_2_ humidified incubator. After 2 days, the medium was changed to NSCs neurogenic differentiation medium (Cat no. RAXNX-90081, Cyagen Biosciences, Suzhou, China). The differentiation medium was replaced every 3 days, and the NSCs were co-cultured with control (DMSO) or bpV(pic)/PLGA microspheres for 3 days. Then the NSCs were analyzed with western blot and immunofluorescence staining.

### Cell survival assay

Cell survival assay was performed with the use of the cell counting kit-8(CCK-8) according to the manufacturer's recommendations (Beyotime Biotechnology, China). Briefly, NSCs were cultured as monolayer in wells of a 96-well culture plate at a cell density of 1 × 10^4^ cells per well. After co-cultured with saline, ASC scaffold only, bpV(pic)/PLGA microspheres only and ASC scaffold incorporated with bpV(pic)/PLGA microspheres for 24 hours, NSCs in all groups were rinsed twice with PBS, and then 10 μL of CCK-8 solution were added to each well. After incubation for 4 h, the cell proliferation was evaluated by measuring the absorbance at 450 nm using a microplate reader.

### Western blot analysis

Tissues and cells were lysed using lysis buffer (62.5 mM Tris–HCl (pH 6.8), 10% glycerol, 2% SDS, 50 mM dithiothreitol, 0.01% bromophenol blue) at 96 °C for 10 min. The samples were separated with SDS-PAGE for 70 min. After electrophoresis, proteins were transferred onto membranes (Bio-Rad Laboratories, USA) using a wet transfer method. Each membrane was then incubated in primary antibodies overnight at 4 °C on a shaker. After incubation in specific secondary antibodies, immunoblots were detected using an enhanced chemiluminescence kit (ECL kit, Proteintech, USA).

### Antibodies

Anti-PTEN (ab32199, Abcam, USA), anti-*p*-PTEN (#9554, Cell Signaling Technology, USA), anti-glial fibrillary acidic protein (ab68428, Abcam), anti-βIII-tubulin (ab78078, Abcam), anti-Nestin (ab6142, Abcam), anti-cyclin-D1 (#2987, Cell Signaling Technology), anti-caspase-3 (ab44976, Abcam), anti-PARP (#9532, Cell Signaling Technology), anti-pS6(s235/236) (#4858, Cell Signaling Technology), anti-S6(#2317, Cell Signaling Technology), anti-pAKT(s473) (#4060, Cell Signaling Technology), anti-AKT (#2920, Cell Signaling Technology), anti-CGRP (#14959, Cell Signaling Technology), anti-β-actin (#3700, Cell Signaling Technology).

### Quantitative reverse transcription-polymerase chain reaction (qRT-PCR)

Total RNA was isolated with Trizol (Life Technologies, USA) and reverse transcription was performed with reverse transcriptase (Takara Bio, Japan) according to the manufacturer's instructions. qRT-PCR was performed using multiple kits (SYBR Premix Ex TAQ, Takara Bio, Japan) according to the manufacturer's instructions. To determine the expression of mRNA, each gene was normalized to the expression level of the housekeeping gene GAPDH. The primers used in the present study are listed below:

PTEN, forward: 5-CAA GAT GAT GTT TGA AAC TAT TCC AAT G-3;

PTEN reverse: 5-CCT TTA GCT GGC AGA CCA CAA-3;

β-III-Tubulin, forward: 5-GAG GGC GAG ATG TAC GAA GA-3;

β-III-Tubulin, reverse: 5-CCT ATG GTG GGA AAA CAG GA-3;

GFAP, forward: 5-CGA GTT ACC AGG AGG CAC TA-3;

GFAP, reverse: 5-TCC ACG GTC TTT ACC ACA AT-3;

GALC, forward: 5-CGG CGT TAG TAT TAG CGG TT-3;

GALC, reverse: 5-AAC TTT CGC TCG ACG TTA CC-3;

Nestin, forward: 5-GAG AAC CAG GAG CAA GTG AA-3;

Nestin, reverse: 5-TTT CCA GAG GCT TCA GTG TC-3.

### Rat spinal cord hemi-section model and graft transplantation

Adult male SD rats (body weight 200–250 g) were purchased from the animal center of Youjiang Medical College for Nationalities (Baise, Guangxi, China). All surgical procedures were performed under anesthesia by intraperitoneal injection with 10% chloral hydrate (0.4 ml/100 g). The spinal laminectomy was performed at the T9-10 level, exposing one thoracic spinal cord segment. Under a surgical microscope, two right-sided hemi-sections of the spinal cord were created using a micro-dissection scissor at levels T9 and T10. A gap of 2 mm width was produced, and the tissue was removed with a 22-gauge ethylene tetrafluoroethylene (ETFE) needle.^39^ Animals that underwent a laminectomy without SCI were used as a sham control (*n* = 4). Animals with a hemi-sectioned SCI were randomly divided into 4 groups after SCI: animals treated with an ASC scaffold implantation (*n* = 6), animals treated with implantation of bpV(pic)/PLGA microspheres (*n* = 6), animals treated with the implantation of an ASC scaffold incorporated with bpV(pic)/PLGA microspheres (*n* = 6), and SCI only (*n* = 6). The muscle layers and skin were closed with suture. Animals were returned to their cages with water and food easily accessible. To prevent infection, rats were treated with ampicillin (100 mg kg^−1^) and gentamicin (12 mg kg^−1^) subcutaneously once a day following surgery for 3 days. Manual bladder expression was performed twice a day until they regained bladder control, approximately 3 to 5 days after initial injury. All animal procedures were performed in accordance with the Guidelines for Care and Use of Laboratory Animals of Youjiang Medical College for Nationalities and approved by the Animal Ethics Committee of Youjiang Medical College for Nationalities.

### Behavioral assessment of rats after different treatments following SCI

#### BBB scoring

A behavioral test was performed to measure the functional recovery of rats' hind limb following treatment.^27^ The score of each hind limb was recorded and the averages were determined, and results were scored on a scale of 0 to 21. Individual rats were placed on an open field and observed for 4 min by two observers blind to the treatment condition. The test was carried out once a week after transplantation up to 6 weeks post-surgery.

### Histological analysis

After surgery, animals were deeply anesthetized with an overdose of chloral hydrate, and transcardiacally perfused with 100 ml of heparinized saline, followed by 100 ml of 4% ice-cold paraformaldehyde. The whole spinal column was then dissected into segments and post-fixed in 4% paraformaldehyde overnight. Then, spinal cord segments were cryoprotected in a 30% sucrose solution in PBS. The spinal cord was embedded in OCT mounting media (Sakura Finetek, USA) and cut into 5 μm coronal and horizontal sections using a cryostat. Immunofluorescence was then performed on spinal cord sections. Briefly, each section was washed with PBS and permeabilized with 0.1% Triton X-100 for 5 min, washed with PBS three to five times, then blocked in 10% bovine serum albumin (BSA, Sigma, USA). After blocking, sections were incubated in primary antibody for 24 h at 4 °C. Then, the appropriate secondary antibodies were applied for 60 min at room temperature, and 4,6-diamidino-2-phenylindole (DAPI) (Molecular Probes, USA) was used as a counterstain to visualize nucleated cells. The axon length was analyzed with the NIH ImageJ software as described previously. In summary, the scale bar was firstly calibrated in ImageJ, then the freehand trace tool was used to measure the distance where the CaP motor axons extended from the spinal cord to the most ventral axonal projection. The mean length of axons was measured from at least 5 replicates and was reported ± SD.^28^

### TUNEL staining

Tissues were fixed in formalin, embedded in paraffin, and then stained with TUNEL using the DeadEnd™ Fluorometric TUNEL System (Promega Corporation, USA), according to the manufacturer's instructions. Apoptotic cells were marked in green and nuclei were marked in blue with DAPI.

### Scanning electron microscopy (SEM)

The micro morphology of the bpV(pic)/PLGA microspheres, ASC scaffolds and ASC scaffolds loaded with bpV(pic)/PLGA microspheres was observed using SEM. Samples were dried for 48 h and coated with a thin layer of gold. Then the samples were subjected to SEM observation.

### Statistical analysis

All experiments were performed at least three times. All data are presented as mean ± standard deviation (SD) using SPSS version 20.0 software for statistical analysis, with graphs generated in GraphPad Prism 6.0. A Student's *t*-test was used to assess statistically significant differences in the data between groups. Values of *p* < 0.05 were considered statistically significant.

## Results

### Inhibiting the expression of PTEN promotes NSCs differentiation and axonal growth

To determine the potential role of PTEN in NSC differentiation, the level of PTEN expression during NSC differentiation (NSCs were incubated in neuronal differentiation induction medium (NIM)) was examined from day 0 to day 14, *via* western blot analysis. The expression levels of both β-III-tubulin and PTEN gradually increased (Fig. 1a and b), suggesting that PTEN may play a vital role in NSC differentiation. Next, siRNA was used to knockdown PTEN, as well as the PTEN inhibitor, bpV(pic), in NSC cultures. Western blot analysis revealed that knocking down PTEN in NSCs resulted in an increased β-III-tubulin expression and decreased Nestin expression with NIM treatment for 3 days (Fig. 1c). Similar results were obtained in qPCR analysis (Fig. 1d), where markers of NSC differentiation (including β-III-tubulin, GALC and GFAP genes) were up-regulated, while Nestin and PTEN gene expression were down-regulated. Next, NSCs were stimulated with different concentrations of bpV(pic) for 3 days in NIM. We found that the level of PTEN gradually diminished with increased bpV(pic) concentration. Surprisingly, the expression of β-III-tubulin was also increased with increased bpV(pic) concentration, in which the highest level of β-III-tubulin expression was observed at a bpV(pic) concentration of 20 ng ml^−1^ (Fig. 1e). When NSCs were incubated with both NIM and bpV(pic), β-III-tubulin expression also increased with increasing incubation time, which was examined using western blot analysis (Fig. 1f) and immunofluorescence staining analysis (Fig. 1g and h). These findings indicate that the inhibition of PTEN expression, by siRNA transfection or its inhibitor bpV(pic), is able to promote the differentiation of NSCs and axonal growth *in vitro*.

**Fig. 1:** siRNA-mediated knock-down of PTEN or inhibition of PTEN with bpV(pic) promotes NSC differentiation. (a) Immunoblot analysis of PTEN, β-III-tubulin and β-actin levels in NSCs after incubation with NIM for 0, 1, 3, 5, 7, and 14 days; *n* = 3 independent experiments. (b) Quantification of the levels of PTEN expression from day 0 to 14. *n* = 3 independent experiments. (c) Immunoblot analysis of PTEN, β-III-tubulin, Nestin and β-actin expression in NSCs following transfection with PTEN siRNA or vehicle, stimulated with NIM for 3 days, *n* = 3 independent experiments; (d) the expression levels of PTEN, β-III-tubulin, GFAP, GLAC and Nestin in NSCs as measured by QPCR. NSCs were transfected with PTEN siRNA or vehicle and stimulated with NIM for 3 days, *n* = 3 independent experiments; (e) immunoblot analysis of *p*-PTEN, β-III-tubulin and β-actin in NSCs treated with different concentrations of bpV(pic) (0, 1, 5, 10, 20 or 50 ng ml^−1^) and NIM for 3 days, *n* = 3 independent experiments; (f) immunoblot analysis of *p*-PTEN, β-III-tubulin and β-actin in NSCs treated with vehicle or 20 ng ml^−1^ bpV(pic) and NIM for 1, 3 and 7 days, *n* = 3 independent experiments; (g) representative images of the immunofluorescence staining analysis of β-III-tubulin in NSCs treated with vehicle or 20 ng ml^−1^ bpV(pic) and NIM for 1, 3 days, scale bar = 50 μm; (h) quantification of the average axonal length, *n* = 5, *p < 0.05, **p < 0.01, all data are shown as mean ± SD.

### Fabrication of ASC composite scaffolds for controlled bpV(pic) release

Since bpV(pic) which inhibits PTEN expression promotes the NSCs differentiation into neurons *in vitro*, it could be considered as a potential therapeutic agent to treat SCI, resulting in reduced tissue damage and neuron death, and a promoted functional recovery after SCI such as hemi-section of the spinal cord. To deliver bpV(pic) in a sustained manner, a new strategy was employed. As shown in Fig. 2a, bpV(pic) was first loaded in PLGA microspheres *via* double emulsion technique. And we noticed that PLGA-loaded ASC scaffolds exhibited a slightly slower weight loss than pure ASC scaffolds, which could be attributed to the slow degradation of PLGA particles (Fig. 2b). The as-prepared bpV(pic)/PLGA microspheres were then incorporated in ASC scaffolds to form bpV(pic)/PLGA/ASC composite scaffold, which was further subjected to implantation into the defected site in spinal cord after hemi-section. The loading of bpV(pic) in PLGA could reduce its release rate during incubation or implantation while the ASC scaffold could provide a biomimetic platform for better grafting with host spinal cord tissue. hematoxylin and eosin (H&E) and Masson's trichrome staining of sectioned ASC scaffolds revealed the ASC scaffolds had a bundle-like structure with certain alignment. The immunofluorescence staining of collagen type II confirmed that the scaffold was primarily comprising of collagen (Fig. 2c). The bpV(pic) loaded PLGA microspheres were round in shape and had a diameter of 70–120 μm. The surface of ASC scaffolds was rough, showing a typical hydrogel-like morphology. It is found that bpV(pic) loaded PLGA microspheres were uniformly dispersed in ASC scaffolds (Fig. 2d). The effect of such composite scaffold on neural tissue regeneration and functional recovery was verified in a rat model with laterally hemi-sectioned SCI.

**Fig. 2:** Fabrication of the ASC scaffold with bpV(pic)/PLGA microspheres. (a) Illustrative schematic of fabricating ASC scaffolds incorporated with bpV/PLGA microspheres for regeneration of spinal cord tissue; (b) *in vitro* degradation behaviour of PLGA microspheres and PLGA microsphere-loaded ASC scaffolds. (c) H&E staining, Masson's trichrome staining and immunofluorescence staining with collagen II of the ASC scaffold. Scale bar = 50 μm. (d) Scanning electron microscope structural analysis of the ASC scaffold, bpV(pic)/PLGA microspheres and ASC scaffold incorporated with bpV(pic)/PLGA microspheres.

### bpV(pic)/PLGA microspheres promote axonal growth, enhance NSC proliferation and decrease NSC apoptosis

The release behavior of bpV(pic) from ASC scaffolds embedded with bpV(pic) loaded PLGA microspheres is shown in Fig. 3a. In initial 12 h, rapid bpV(pic) release with a 53% level was obtained, followed by a slow bpV(pic) release up to 60% in 96 h. To evaluate the effect of the bpV(pic)/PLGA microspheres on NSCs, we co-cultured NSCs together with bpV(pic)/PLGA microspheres. After 3 days of stimulation with NIM, when NSCs were incubated with bpV(pic)/PLGA microspheres., longer axons and neurites can be observed, compared to that of the control group (Fig. 3b and e). The survival rate of NSCs were not affected in comparison with the control group (Fig. 3c). The expression of β-III-tubulin in NSCs was then studied *via* immunofluorescence staining. Consistent with results obtained in Fig. 3b, incubating NSCs with bpV(pic)/PLGA microspheres resulted in higher β-III-tubulin expression by showing longer axon length, compared to control groups (Fig. 3d). Afterwards, proteins were extracted from the stimulated cells for western blot analysis. Compared to the control groups, bpV(pic)/PLGA group induced higher level of β-III-tubulin and GFAP (astrocytic marker) and lower level of Nestin (stem cell marker) (Fig. 3f). Besides, bpV(pic)/PLGA group decreased the expression level of apoptosis related proteins (PARP and caspse-3), but up-regulated the proliferation marker, cyclin D1 (Fig. 3g). These data demonstrate that bpV(pic) loaded microspheres promoted axonal growth, enhanced proliferation and decreased apoptosis in NSCs *in vitro*.

**Fig. 3:** Assessing the effect of bpV(pic)/PLGA on NSCs *in vitro*. (a) Release curve of bpV(pic)/PLGA microspheres *in vitro*; (b) NSCs were cultured for 3 days under the following different conditions: NIM with DMSO, NIM plus bpV(pic)/PLGA, representative images of the treated NSCs are shown, scale bar = 50 μm; (c) NSCs were co-cultured with DMSO or bpV(pic)/PLGA microspheres for 24 hours, and then cell survival was analyzed by CCK-8 assay, *n* = 3 independent experiments, ns = not significant, all data are shown as mean ± SD; (d) immunofluorescence analysis of β-III-tubulin expression in NSCs after treatment with NIM with DMSO and NIM plus bpV(pic)/PLGA for 3 days. Scale bar = 50 μm; (e) quantification of the average axonal length from differentiated NSCs cultured under different conditions. *n* = 5; (f) immunoblot analysis of β-III-tubulin, GFAP, Nestin and β-actin levels in NSCs cultured under different conditions, *n* = 3 independent experiments; (g) immunoblot analysis of PARP, caspase-3, cyclin-D1 and β-actin levels in NSCs cultured under different conditions, *n* = 3 independent experiments. ns = not significant, **p < 0.01. All data are shown as mean ± SD.

### ASC scaffolds incorporated with bpV(pic)/PLGA microspheres improve axonal regeneration and functional recovery in a rat model of spinal cord injury

We next assessed the efficacy of the ASC scaffolds incorporated with bpV(pic)/PLGA microspheres on the treatment of a rat model with hemi-sectioned SCI. At 4 weeks post-surgery, spinal cord tissue was harvested, and the general appearance of the spinal cords grafted with ASC scaffold, bpV(pic) and bpV(pic)/PLGA/ASC scaffold was shown in Fig. 4a. The motor function of animals from different groups was measured using the BBB (Basso–Beattie–Bresnahan score) system. The ASC-only treated group showed comparable BBB scores with the control group, whereas the bpV(pic)/PLGA group showed a significant improvement in score (*p* < 0.05). The ASC scaffold incorporated with bpV(pic)/PLGA microspheres group had the extraordinarily significantly improved BBB score (Fig. 4b). The spinal cord tissues treated with different agents were then sectioned and processed for H&E staining. As shown in Fig. 4c, the tissue in the lesion zone was badly disrupted in control and ASC-only groups, showing cavities with varied size, while the lesion gap was partially covered in the bpV(pic)/PLGA group, and was completely fused in the ASC scaffold incorporated with bpV(pic)/PLGA microspheres group. We also determined the expression levels of *p*-PTEN and β-III-tubulin in the regenerated tissues collected from all groups by immunofluorescence staining. The expression of phosphorylate PTEN was down-regulated in the bpV(pic)/PLGA and ASC scaffold incorporated with bpV(pic)/PLGA microspheres groups (Fig. 4d). As expected, the expression of β-III-tubulin was increased in the bpV(pic)/PLGA group, the axons grew along and extended into the implant and greatly increased in the ASC scaffold incorporated with bpV(pic)/PLGA microspheres group (Fig. 4). We also performed immunofluorescence staining of calcitonin gene-related peptide (CGRP) to trace axonal re-growth through the site of injury, and found that the ASC scaffold combined with bpV(pic)/PLGA microspheres group had the highest level of re-growth compared to all other treatment groups (Fig. 4e). Finally, we noticed that the number of TUNEL and GFAP positive cells was diminished in the bpV(pic)/PLGA and ASC scaffold incorporated with bpV(pic)/PLGA microspheres groups compared to control and ASC-only groups (Fig. 4f and g), suggesting the number of apoptosis cells and astrocytes in the bpV(pic)/PLGA and ASC scaffold group was significantly decreased. These results demonstrate that the sustained release of bpV(pic) from PLGA microspheres and the presence of biomimetic ASC scaffolds in the spinal cord with SCI could improve axonal regeneration and functional recovery.

**Fig. 4:** An ASC scaffold with bpV(pic)/PLGA microspheres improves SCI recovery *in vivo*. (a) Gross appearance of the spinal cord grafted with control, ASC, bpV(pic)/PLGA and the ASC scaffold with bpV(pic)/PLGA microspheres; (b) plot of BBB locomotor scores of the different transplantation groups at different times (from 1 to 6 weeks) post-SCI, *n* = 6; (c) H&E staining of spinal cords from SCI rats 4 weeks post-surgery from the following experimental conditions: no graft, ASC-only graft, bpV(pic)/PLGA-only graft, or ASC scaffold with bpV(pic)/PLGA graft. Scale bar = 50 μm; (d) representative immunofluorescence images and quantification of the number of *p*-PTEN (green) and β-III-tubulin (red) staining in the lesion part of the spinal cords from SCI rats with no graft, ASC-only graft, bpV(pic)/PLGA-only graft or ASC scaffold with bpV(pic)/PLGA graft at 4 weeks post-surgery. *n* = 6, scale bar = 50 μm; (e) representative immunofluorescence images and quantification of the number of CGRP fibers in the lesion part of spinal cord of SCI rats with different treatments. *n* = 6, scale bar = 50 μm; (f) TUNEL analysis of the apoptotic cells in the lesion part of the spinal cord of SCI rats with different treatments. *n* = 6, scale bar = 50 μm; (g) representative immunofluorescence images and quantification of the number of GFAP in the lesion part of the spinal cord of SCI rats with different treatments. C represents the lesion cavity. *n* = 6, scale bar = 50 μm; *p < 0.05, **p < 0.01. All data are shown as mean ± SD.

### bpV(pic) treatment improves axonal regeneration post-injury by activating the AKT–mTORC1 pathway

Several studies reported that the AKT–mTOR pathway promotes neuroprotection following trauma and in CNS disease. Given that PTEN is a key modulator of AKT–mTOR signaling, we hypothesized that the therapeutic effect of the PTEN inhibitor bpV(pic) on axonal regeneration post-SCI may act *via* regulation of the mTOR pathway. To explore this possibility, we evaluated the progression of mTORC1 signaling during the NSC differentiation process. As shown in Fig. 5a and d, the expression level of the mTORC1 downstream effector protein, pS6(s235/236), decreased while the level of β-III-tubulin increased during differentiation (*i.e.*, day 0 to 7), during which PTEN expression gradually increased. By western blot analysis, the expression level of β-III-tubulin increased gradually during the period of NIM incubation from days 0 to 14, while Nestin, *p*-AKT and pS6 levels decreased (Fig. 5b). We also noticed a reduced level of pS6 in spinal cords *in vivo* when the SCI exacerbated (*i.e.*, 2, 4 and 8 weeks following cervical hemi-contusion surgery, Fig. 5c and e). Thus, we speculate that the PTEN–AKT–mTOR pathway may participate in the process of NSC differentiation following SCI.

**Fig. 5:** bpV(pic) treatment improves axonal regeneration after SCI by activating AKT–mTORC1. (a) Representative immunofluorescence images of pS6 (green) and β-III-tubulin (red) staining in NSCs after incubation with NIM for 0, 3 and 7 days. Scale bar = 50 μm; (b) immunoblot analysis of *p*-AKT(s473), AKT, pS6(s235/236), S6, β-III-tubulin, Nestin and β-actin levels in NSCs after incubation with NIM for 0–14 days, *n* = 3, independent experiments; (c) representative immunofluorescence images of pS6 (green) staining in the lesion part of spinal cords from normal rats and SCI rats at 2, 4 and 8 weeks post-surgery. Scale bar = 50 μm; (d) quantification of the number of pS6 (green) positive cells, *n* = 5, *p < 0.05, all data are shown as mean ± SD; (e) quantification of the number of pS6 (green) positive cells, *n* = 5, *p < 0.05, all data are shown as mean ± SD; (f) representative immunofluorescence images of pS6 (green) and β-III-tubulin (red) staining in the lesion part of spinal cords from SCI rats with no graft, ASC-only graft, bpV(pic)/PLGA-only graft or ASC scaffold with bpV(pic)/PLGA graft at 4 weeks post-surgery, C represents the lesion cavity. Scale bar = 50 μm; (g) quantification of the number of pS6 (green) positive cells, *n* = 6, ns = not significant, *p < 0.05, **p < 0.01, all data are shown as mean ± SD; (h) immunoblot analysis of *p*-PTEN, pS6, S6, *p*-AKT, AKT and β-actin levels in the spinal cord of SCI rats with no graft, ASC-only graft, bpV(pic)/PLGA-only graft or ASC scaffold with bpV(pic)/PLGA graft at 4 weeks post-surgery., *n* = 3 independent experiments; (i) immunoblot analysis of β-III-tubulin, GFAP, PARP, caspase-3, pS6, S6, *p*-AKT, AKT and β-actin levels in NSCs after treatment with vehicle, bpV(pic), bpV(pic) plus rapamycin and bpV(pic) plus LY294002 for 24 hours, *n* = 3 independent experiments.

We finally sought to confirm whether the administration of bpV(pic) acts through PTEN inhibition and subsequent upregulation of mTOR activity *in vivo*. We examined the activity of mTORC1 signaling in rats following SCI surgery from each group. As determined by immunofluorescence and western blot analyses, the expression levels of pS6 and *p*-AKT were increased in the bpV(pic)/PLGA and ASC scaffold incorporated with bpV(pic)/PLGA microspheres groups as the levels of β-III-tubulin increased (Fig. 5f–h). In cultured NSCs, stimulation with bpV(pic) enhanced the expression of the differentiation markers β-III-tubulin and GFAP, while also decreasing levels of apoptotic markers caspase-3 and PARP (Fig. 5i). Combining bpV(pic) treatment with the mTORC1 inhibitor rapamycin or AKT–PI3K inhibitor LY294002 was sufficient to reverse these effects (Fig. 5i). Thus, it is reasonable to think that bpV(pic) treatment improves axonal regeneration post-injury by activating the AKT–mTORC1 pathway.

## Discussion

Due to extensive neuronal loss, acute axonal damage and demyelination, SCI often results in severe sensory and motor neuron deficits.^8,29^ After CNS injury such as SCI, limited axonal re-growth *in vivo* is often obtained due to a reduced growth capacity of mature axons.^30^ A growing number of investigators are pushing their way through discovering new approaches for spinal cord regeneration, including molecular and cellular approaches and implanted neuro-prosthetic device, and some of which showed potential therapeutic treatment for SCI with ability to promote axon regeneration and restore functional motor.^31–33^ Several studies have demonstrated that the treatment with the PTEN phosphatase inhibitor, bpV(pic), could reduce neural tissue damage/neuron death and promote functional recovery, following a hemi-sectioned SCI.^23,24^ The present study combined an ASC scaffold with bpV(pic)/PLGA microspheres to treat SCI in a rat model with hemi-section of the spinal cord. The bpV(pic)/PLGA microspheres showed excellent biocompatibility and improved capability to promote axonal growth *in vitro.* In the treatment of rat SCI *in vivo*, an ASC scaffold was used to load bpV(pic)/PLGA microspheres and the implantation of the composite scaffolds in defected spinal cord resulted in improved axonal regeneration and functional recovery *in vivo* compared to treatment of ASC scaffolds or bpV(pic)/PLGA microspheres alone. We also determined that bpV(pic) likely functions by inhibiting the phosphorylation of PTEN, thereby resulting in substantial activation of the mTORC1/AKT pathway. Importantly, activation of the mTORC1/AKT pathway by bpV(pic) treatment resulted in decreased apoptosis,^34^ increased proliferation and increased axonal growth both *in vitro* and *in vivo*.^35–37^ Due to all these effects, bpV(pic) was able to promote neuroprotection and ameliorate the SCI recovery process. We have, therefore, successfully constructed a new structure which combines an ASC scaffold with a controlled release of bpV(pic), thereby greatly improving the effectiveness of bpV(pic) in the treatment of SCI.

Previous studies shown that PI3K–AKT–mTOR pathway controls the axonal elongation and also regulates cell survival, growth, proliferation and differentiation.^38,39^ Since PTEN is a natural inhibitor of the PI3K/AKT pathway, the inhibition of PTEN activity could temporarily and safely affect the PI3K/AKT pathway and activate mTOR signaling, thereby influencing cell survival, proliferation and migration. bpV(pic) is a specific inhibitor of PTEN's phosphatase activity and has a definite half-life. In our study, the sustained delivery of bpV(pic) to NSCs *in vitro* continuously enhanced the mTORC1 signaling and an increased capacity for neuron differentiation was observed. The addition of rapamycin, a specific inhibitor of mTORC1, together with bpV(pic), resulted in a reversal of the decreased apoptosis and increased differentiation caused by bpV(pic), which was in agreement with previous findings in which bpV(pic) promoted neural regeneration *via* inhibiting PTEN.

Towards the regeneration of the defected spinal cord tissue, finding a suitable tissue engineering scaffolds is highly important. Our previous study showed that an ASC scaffold, seeded with human umbilical cord blood-derived mesenchymal stem cells, was able to bridge a spinal cord cavity and promote long-distance axonal regeneration and functional recovery following SCI.^40^ In the present study, ASC scaffold derived from rat spinal cords was used as an excellent platform for inducing spinal cord tissue regeneration. Combining the ASC scaffold with bpV(pic)/PLGA microspheres resulted in not only an enhanced promotion of NSC differentiation *in vitro* compared to treatment with bpV(pic)/PLGA microspheres alone, but also an increase in NSC differentiation *in vivo*, which is a critical component of the neuroprotective response following SCI. We believe that the activation of the mTOR pathway by bpV(pic)/PLGA microspheres, combined with the physical contact of an ASC scaffold, led to the regenerative effects observed.

In summary, composite neural tissue engineering scaffold consisting of an ASC scaffold and bpV(pic)/PLGA microspheres was successfully constructed. Controlled release of bpV(pic) promoted NSC differentiation and decreased the NSC apoptosis *in vitro*. Implanting the composite scaffold into a hemi-sectioned spinal cord induced improved tissue regeneration and improved the locomotor function of animals, providing a neurotrophic, protective effect and changing the lesion microenvironment in order to help host cells to regenerate.

## Author contributions

Y. J. T. conceived the project, designed and supervised the experiments, and wrote the manuscript. C. W., K. L. and J. L. performed the experiments and analyzed the data. Y. H. W., K. H., T. S. and Z. P. H. helped with the animal and cell-cultured experiments. Y. P. H., J. Z. and Q. S. L. helped prepare the figures and finished the IHC/IF and WB analysis.

## Conflicts of interest

The authors have no conflicts of interest to declare.

## Funding statement

This work was supported by the National Natural Science Foundation of China (81560213 and 81760450), Natural Science Foundation of GuangXi (2018GXNSFAA138074) and supported by Chongqing Postdoctoral Research Special Fund (Xm2017181).

## Supplementary Material
